# The Simplified Analytical Algorithm to the Time Effect of the Simple-Supported Steel and Concrete Composite Beam

**DOI:** 10.1155/2022/4951080

**Published:** 2022-08-17

**Authors:** Kai-cheng Yao, Dong-hua Zhou, Yingcheng He, Shilong Wu

**Affiliations:** ^1^School of Construction Engineering, Kunming University of Science and Technology, Kunming 650504, China; ^2^Kunming Engineering & Research Institute of Nonferrous Metallurgy Co., Ltd., Kunming 650504, China

## Abstract

Based on Rusch's creep constitutive relation, differential equations for the redistribution of shrinkage internal force and creep of the composite beam are derived and solved. The closed solution is cumbersome and is inconvenient to be applied practically. It is hard to solve the accurate solution for coupled differential equations. Therefore, a simplified approach is given. However, it ignores the influence of the redistribution of bending moment of the concrete slab on the axial strain and removes the coupling relationship of differential equations so that it makes the solution become convenient. The comparison of the results calculated by the two approaches shows that their calculated errors are small, within 3%, when the stiffness ratio of the concrete slab and the steel beam are less than 0.185. It also shows that the greater the stiffness of the steel beam, the greater the constraint on the creep of the concrete slab, so is the redistribution of internal force.

## 1. Introduction

Steel-concrete composite beam (hereinafter referred to as “composite beam”) is a member compounded by shape steel and concrete slab through shear joints [1] with good bearing capacity, rigidity, and constructive performance, which is used more and more extensively [2]. The concrete slab in the composite beam has long-term effects that are the shrinkage and creep. However, there are no shrinkage or creeping effects for the steel beam. Therefore, along with changes in time, the interaction force will be generated between the steel beam and the concrete slab, leading to the redistribution of internal force of the composite beam. The redistribution of internal force is a factor that must be considered while the composite beam is designed. The support condition of the composite beam will affect the initial internal force of the section of the composite beam and the internal force of the full section. In this paper, the composite beam (the simple structure) under the condition of simple support is studied. Effects of shrinkage and creep of the concrete slab only cause the internal force to be generated inside some sections, such as the concrete slab and the steel beam, and the internal force of the full section of the composite beam cannot be changed [3–5].

Based on Rusch's creep constitutive equation, this paper deduces the analytical exact solution equation of the redistributed internal force of the composite beam. In order to make the calculation formula more concise and more suitable for engineering practice, the simplified analytical equation is rederived by ignoring the effect of redistributed bending moment in the concrete slab on the axial strain. Finally, it is proved that the accuracy of the simplified method can meet the requirements of use through an example.

## 2. Constitutive Relation and Basic Assumptions

### 2.1. Constitutive Relation

The creep constitutive relation is the basis for calculating the effect of creep. Different creep constitutive relations lead to different methods of calculation. Dischinger proposed the relationship of creep time [6] (see Figure 1(a)) that the creep rate and loading age are irrelevant. The creep curve of the subsequent loading can be obtained by moving the initially loaded creep curve downward in parallel, thereby making the integral constitutive equation be transformed into the differential constitutive equation, which is called the rate of the creep method [7–9]. However, Dischinger's creep constitutive equation does not contain hysteresis elastic deformation. All of these creep deformations are plastic deformations. And it is quite different from the actual measured results. In order to overcome this deficiency, Rusch improved Dischinger's relationship of creep time and decomposed the creep coefficient into two, which are the plasticity strain that is creep plasticity and deformation and hysteresis elastic strain that is the hysteresis elastic deformation (see Figure 1(b)). The creep constitutive equation obtained thereout is called the improved Dischinger method, and the result obtained by Rusch's constitutive equation is closer to the reality.

### 2.2. Basic Assumptions and Symbolic Rules

Results obtained from a large number of tests and numerical calculations have proved that both the steel beam and the concrete slab are in the elastic working stage under the normal use of composite beam [5, 10, 11]. At the same time, the following assumptions are made to simplify the process of calculation and analysis:

  (1) The bending moment and axial force of the member do not change as the change of time.
  (2) The slip between the concrete slab and the steel beam is neglected.
  (3) The sectional deformation of the composite beam satisfies the assumption for flat section.
  (4) The crack of the concrete slab is not considered.
  (5) It is assumed that the process of shrinkage is the same as that of creep.
  (6) The influence of reinforcement steel bar is ignored in the analysis of creep.

For the convenience of calculation, the plus sign and minus sign in this paper are defined as follows: (1) in terms of the deformation, the plus sign is for the internal force, so is the corresponding deformation, and vice versa; (2) in terms of the internal force, the plus sign is for the axial force making the member be pulled, so is the bending moment making the bottom of beam be pulled, and vice versa.

## 3. The Analysis for the Accurate Algorithm (Exact Method)

Under the premise of basic assumptions, the exact method is to incorporate all parameters into the calculation and can obtain relatively accurate calculation results, which is suitable for most situations. The disadvantage is that the calculation process is cumbersome and not suitable for hand calculation. In this paper, the Lüxiu constitutive relation is used to calculate the internal force redistribution of composite beams accurately.

Rusch's creep constitutive equation is as follows:

(1) $$\begin{array}{c} d\varepsilon \left(t\right)=\frac{1}{E}d\sigma \left(t\right)\left(1+\varphi_{d}\right)+\frac{1}{E}d\sigma \left(t\right)d\varphi_{f}\left(t\right)+d\varepsilon_{sh}\left(t\right), \end{array}$$

where *φ*_*f*_=*φ*_*t*_ − *φ*_*d*_, where *φ*_*t*_ are creep coefficients, *φ*_*f*_ is the plastic creep coefficient, and *φ*_*d*_ is the hysteretic elastic creep coefficient, and the final value is 0.4. In Rusch's method, only the creep plasticity and creep deformation change with the change in time, and the hysteretic elastic strain can take the final value and be superimposed with the elastic strain.

When the creep problem of the composite beam is solved, the internal force at three moments (see Figure 2), *t*_0_ (before creep), *t* (any moment after creep), and the internal force (the time increment at the *t* moment), need to be considered. There is initial internal force *M*_0_ and *N*_0_ on the section at *t*_0_ moment, which includes the initial internal force *M*_*c*0_, *dt*, and *N*_*c*0_ on the section of concrete slab (I represents the concrete slab) and the initial internal force *M*_*s*0_ and *N*_*s*0_ on the section of steel beam (*s* represents the steel beam). Due to the shrinkage and creep at the *t* moment, the redistribution of internal force *M*_*cr*_, *N*_*cr*_, *M*_*sr*_, and *N*_*sr*_ inside the section occurs, which is self-phase balanced and is the unknown to be sought. The increments for the redistribution of internal force are *dM*_*cr*_, *dN*_*cr*_, *dM*_*sr*_, and *dN*_*sr*_. The internal force of the full section at the *t*_0_ moment can be distributed according to the stiffness, which is carried out as

(2) $$\begin{array}{c} \left.\begin{array}{c} N_{c0}=\frac{A_{cr}}{A_{i}}N_{0}-\frac{S_{i}}{I_{i}}M_{0},\;M_{c0}=\frac{I_{cr}}{I_{i}}M_{0}\\ N_{s0}=\frac{A_{s}}{A_{i}}N_{0}+\frac{S_{i}}{I_{i}}M_{0},\;M_{s0}=\frac{I_{s}}{I_{i}}M_{0} \end{array}\right\}. \end{array}$$

The parameters in the equation are *A*_*cr*_=*A*_*c*_/*n*, *I*_*cr*_=*I*_*c*_/*n*, *n*=*E*_*s*_/*E*_*cd*_, *E*_*cd*_=*E*_*c*_/1+*φ*_*d*_, *I*_*i*_=*I*_*cr*_+*I*_*s*_+*S*_*i*_*d*, *A*_*i*_=*A*_*cr*_+*A*_*s*_, and *S*_*i*_=*A*_*s*_*A*_*cr*_/*A*_*s*_+*A*_*cr*_*d*.

The redistribution of internal force at the *t* moment is self-phase balanced. Equations (3) can be obtained thereout as

(3) $$\begin{array}{c} \left.N_{cr}=-N_{sr}-M_{cr}+N_{cr}\cdot d=M_{sr}\right\}. \end{array}$$

The increment for the redistribution of internal force occurred within the time increment *dt* is also self-phase balanced, and incremental equations can be obtained as

(4) $$\begin{array}{c} \left.dN_{cr}=-dN_{sr}-dM_{cr}+dN_{cr}\cdot d=dM_{sr}\right\}. \end{array}$$

Because there are four unknown parameters *M*_*cr*_, *N*_*cr*_, *M*_*sr*_, and *N*_*sr*_ to be solved, four equations need to be found. Only relying on existing equations (3) and (4) cannot meet requirements for the solution so that two equilibrium equations need to be found. According to the assumption that the sectional deformation of the composite beam meets the flat section, two deformation-coordination [12–14] equilibrium equations can be found, in which the strain increment [15–17] and the curvature increment [18, 19] for the steel beam and the concrete slab are equal at any fiber:

(5a) $$\begin{array}{c} \left.\begin{array}{c} d\varepsilon_{c}\left(t\right)=d\varepsilon_{s}\left(t\right)\\ d\phi_{c}\left(t\right)=d\phi_{s}\left(t\right) \end{array}\right\}. \end{array}$$

Equation (5a) is the deformation-coordination equilibrium equation of the strain increment, which is developed at the core of the concrete slab. The left side of the equation is the total strain increment for the concrete slab, including the free strain that is caused by the initial force of the section and constrained strain which is caused by the redistribution of internal force [20–22]. Equation (5b) can be obtained according to Figure 2. The right side of the equation is the total strain increment for the steel beam which is composed by elastic strain only. Equation (5c) can be obtained according to Figure 2. The second equation (5a) is the deformation-coordination equation of curvature increment. Its composite method is similar to the composition of the first equation. Refer to Equations (5d) and (5e).

(5b) $$\begin{array}{c} d\varepsilon_{c}\left(t\right)=1+2+3+4\\ =\frac{\varepsilon_{sh}}{\varphi_{c\infty }}d\varphi_{f,d}+\frac{N_{c0}}{E_{cd}A_{c}}d\varphi_{f,d}+\frac{N_{cr}}{E_{cd}A_{c}}d\varphi_{f,d}+\frac{dN_{cr}}{E_{cd}A_{c}}. \end{array}$$

In the equation, *ε*_*sh*_ is the final value of shrinkage strain and *φ*_*c∞*_ is the final value of creep strain.

(5c) $$\begin{array}{c} d\varepsilon_{s}\left(t\right)=5-6=\frac{dN_{sr}}{E_{s}A_{s}}-\frac{dM_{sr}}{E_{s}I_{s}}d, \end{array}$$

(5d) $$\begin{array}{c} d\phi_{c}\left(t\right)=\left(\text{I}\right)+\left(\text{II}\right)+\left(\text{III}\right) \end{array}$$

(5e) $$\begin{array}{c} d\phi_{s}\left(t\right)=\left(\text{IV}\right)\\ =\frac{dM_{sr}}{E_{s}I_{s}}. \end{array}$$

Substituting Equations (5b)∼ (5d) into Equation (5a), we obtain

(5f) $$\begin{array}{c} \left\{\begin{array}{c} \frac{\varepsilon_{sh}}{\varphi_{c\infty }}d\varphi_{f,d}+\frac{N_{c0}}{E_{cd}A_{c}}d\varphi_{f,d}+\frac{N_{cr}}{E_{cd}A_{c}}d\varphi_{f,d}+\frac{dN_{cr}}{E_{cd}A_{c}}=\frac{dN_{sr}}{E_{s}A_{s}}-\frac{dM_{sr}}{E_{s}I_{s}}d,\\ \frac{M_{c0}}{E_{cd}I_{c}}d\varphi_{f,d}+\frac{M_{cr}}{E_{cd}I_{c}}d\varphi_{f,d}+\frac{dM_{cr}}{E_{cd}I_{c}}=\frac{dM_{sr}}{E_{s}I_{s}}. \end{array}\right. \end{array}$$

In Equation (5b), four unknown parameters *N*_*cr*_, *M*_*cr*_, *N*_*sr*_, and *M*_*sr*_ are contained. *N*_*cr*_, *N*_*sr*_, *dN*_*cr*_, and *dN*_*sr*_ in the equilibrium equations (3) and (4) are substituted into Equation (5b). The differential equations (6) can be obtained after the arrangement. The equations contain only two unknowns *M*_*cr*_ and *M*_*sr*_:

(6) $$\begin{array}{c} \left\{\begin{array}{c} \frac{A_{i}}{A_{s}}\cdot \frac{dM_{cr}}{d\varphi_{f,d}}+M_{cr}+\frac{A_{i}\left(I_{s}+S_{i}d\right)}{A_{s}I_{s}}\cdot \frac{dM_{sr}}{d\varphi_{f,d}}+M_{sr}=-\left(N_{sh}+N_{c0}\right)d,\\ \frac{dM_{cr}}{d\varphi_{f,d}}+M_{cr}-\frac{I_{cr}}{I_{s}}\cdot \frac{dM_{sr}}{d\varphi_{f,d}}=-M_{c0}. \end{array}\right.. \end{array}$$

In the equation, *N*_*sh*_=*ε*_*sh*_/*φ*_*c∞*_*E*_*s*_*A*_*cr*_. The solution of equation (6) can be obtained from the initial condition *t*=0, *φ*_*f*,*d*_=0, and *M*_*cr*_=*M*_*sr*_=0:

(7) $$\begin{array}{c} M_{cr}=-M_{c0}\left\{1+\frac{\rho a_{s}}{\gamma_{1}-\gamma_{2}}\left[\begin{array}{c} \frac{\gamma_{1}\left(1+\rho \right)+1}{\rho \gamma_{1}}e^{\gamma_{2}\varphi_{f,d}}\\ -\frac{\gamma_{2}\left(1+\rho \right)+1}{\rho \gamma_{2}}e^{\gamma_{1}\varphi_{f,d}} \end{array}\right]\right\}-\left(N_{sh}+N_{c0}\right)d\frac{\rho a_{s}}{\gamma_{1}-\gamma_{2}}\left(e^{\gamma_{1}\varphi_{f,d}}-e^{\gamma_{2}\varphi_{f,d}}\right), \end{array}$$

(8) $$\begin{array}{c} M_{sr}=M_{c0}\left\{1+\left[\begin{array}{c} \frac{\left(\gamma_{2}+a_{s}\right)}{\gamma_{1}-\gamma_{2}}\frac{\gamma_{2}\left(1+\rho \right)+1}{\rho \gamma_{2}}e^{\gamma_{1}\varphi_{f,d}}\\ -\frac{\left(\gamma_{1}+a_{s}\right)}{\gamma_{1}-\gamma_{2}}\frac{\gamma_{1}\left(1+\rho \right)+1}{\rho \gamma_{1}}e^{\gamma_{2}\varphi_{f,d}} \end{array}\right]\right\}-\left(N_{sh}+N_{c0}\right)d\left\{1+\left[\begin{array}{c} \frac{\left(\gamma_{2}+a_{s}\right)}{\gamma_{1}-\gamma_{2}}e^{\gamma_{1}\varphi_{f,d}}\\ -\frac{\left(\gamma_{1}+a_{s}\right)}{\gamma_{1}-\gamma_{2}}e^{\gamma_{2}\varphi_{f,d}} \end{array}\right]\right\}, \end{array}$$

(9) $$\begin{array}{c} N_{cr}=N_{sr}=\frac{M_{cr}+M_{sr}}{d}. \end{array}$$

Parameters in the equation are $\gamma_{1,2}=1/2\left[-\left(1+\alpha_{s}-\alpha_{c}\right)\pm \sqrt{{\left(1+\alpha_{s}-\alpha_{c}\right)}^{2}-4\alpha_{s}}\right]$, *α*_*s*_=*A*_*s*_*I*_*s*_/*A*_*i*_*I*_*i*_, and *α*_*c*_=*A*_*cr*_*I*_*cr*_/*A*_*i*_*I*_*i*_, *ρ*=*I*_*cr*_/*I*_*i*_.

It can be seen that equations (7) and (8) are too prolix and inconvenient to use so that a simplified method of calculation need to be found. In addition, it is relatively difficult to solve the coupled differential equations above. If the differential equations can be decoupled [23, 24], the solution will be much easier. The approach to the simplified approximation is described in the following.

## 4. Simplified Method

Because the calculation process of the exact method is very cumbersome, this method is not easy to apply. Under the premise of satisfying the necessary accuracy, in order to improve the calculation efficiency, the precise calculation process can be simplified. The simplification method is based on the exact method, ignoring individual parameters that have little influence on the calculation results so that the calculation process is simplified to the greatest extent.

The following equation can be obtained by substituting the second equation of Equation (4) into Equation (5f):

(10) $$\begin{array}{c} \frac{dN_{cr}}{d\varphi_{f,d}}\left(\frac{1}{E_{cd}A_{c}}+\frac{1}{E_{s}A_{s}}+\frac{d^{2}}{E_{s}I_{s}}\right)+\frac{N_{cr}}{E_{cd}A_{c}}+\frac{N_{c0}}{E_{cd}A_{c}}+\frac{\varepsilon_{c\infty }}{\varphi_{c\infty }}-\frac{dM_{cr}}{d\varphi_{f,d}}\cdot \frac{d}{E_{s}I_{s}}=0. \end{array}$$

The thickness of the concrete slab in the composite beam is much smaller than the height of the steel beam usually, which is more obvious in the bridge. Therefore, compared to the steel beam, the concrete slab has a small antibending rigidity so that the redistribution of bending moment *M*_*cr*_ will be small. Equation (10) contains two unknown functions *N*_*cr*_ and *M*_*cr*_. Its last one item is the axial deformation caused by *dM*_*cr*_ (the increment for *M*_*cr*_ in *d*_*t*_) with small axial strain. In order to simplify equation (10), please ignore this item in the process of calculation so that you can obtain

(11) $$\begin{array}{c} \frac{dN_{cr}}{d\varphi_{f,d}}\left(1+\frac{E_{cd}A_{c}}{E_{s}A_{s}}+\frac{E_{cd}A_{c}d^{2}}{E_{s}I_{s}}\right)+N_{cr}+N_{c0}+N_{sh}=0. \end{array}$$

Now, equation (11) contains one unknown function only, which can be solved independently. The solution for differential equation (9) can be obtained from the initial conditions, *t*=0, *φ*_*f*,*d*_=0, and *N*_*cr*_=0:

(12) $$\begin{array}{c} N_{cr}=\left(N_{sh}+N_{c0}\right)\left(e^{-\left(a_{s}/a\right)\varphi_{f,d}}-1\right), \end{array}$$

where *α*=*I*_*i*_ − *I*_*cr*_/*I*_*i*_.

The derivation operation for *N*_*cr*_ solved is performed, substituted into the second equation of equations (4), and then connected with the second equation of equations (5c) so that the following equation can be obtained:

(13) $$\begin{array}{c} \frac{dM_{cr}}{d\varphi_{f,d}}\left(1+\frac{I_{cr}}{I_{s}}\right)+M_{cr}+\frac{\alpha_{s}}{a}e^{-\left(\alpha_{s}/a\right)\varphi_{f,d}}\frac{I_{cr}}{I_{s}}d\left(N_{sh}+N_{c0}\right)+M_{c0}=0. \end{array}$$

Equation (11) also becomes a differential equation that can be solved independently with only one unknown function. The corresponding solution can be obtained below from the initial conditions, *t*=0, *φ*_*f*,*d*_=0, and *M*_*cr*_=0:

(14) $$\begin{array}{c} M_{cr}=M_{c0}\left(e^{-a_{M}\varphi_{f,d}}-1\right)+\frac{A_{s}I_{cr}d\left(N_{c0}+N_{sh}\right)\left(e^{-a_{N}\varphi_{f,d}}-e^{-a_{M}\varphi_{f,d}}\right)}{A_{i}\left(I_{cr}-I_{i}\right)+A_{s}\left(I_{cr}+I_{s}\right)}, \end{array}$$

where *α*_*N*_=*A*_*s*_*I*_*s*_/*A*_*i*_(*I*_*i*_ − *I*_*cr*_) and *α*_*M*_=*I*_*s*_/*I*_*s*_+*I*_*cr*_.

Now, two unknowns *N*_*cr*_ and *M*_*cr*_ in the concrete slab have been solved and then are substituted into equation (3) so that the two unknowns *N*_*cr*_ and *M*_*cr*_ in the steel beam can be solved. So far, four unknowns for the redistribution internal force of the composite beam have been solved with the simplified method.

Simplifications made in the process of calculation will inevitably cause the error for the result of the calculation. How big is the error? Is there any change regularities in the error? Tests and analysis can be performed by some examples.

## 5. Example

In order to obtain the internal regularities, some examples were selected, which are eight combined sections in Figure 3 with different heights of steal beams. The initial internal force on the full section is *M*_0_ = 2.0*∗*10^3^ kNm, *N*_0_ = 0, *φ*_*t*_ = 4.0, *φ*_*d*_ = 0.4, *φ*_*f*,*d*_ = 2.57, and other parameters which are shown in Figure 3.

The detailed parameters of eight sections are shown in Table 1.  Table 2 shows the initial internal force, the redistribution of internal force (with accurate method and simplified method), and the final internal force of eight sections. It can be observed in the combination of Table 1 that if the stiffness of the steel beam (under the axial direction and bending) increases, so does the redistributed internal force of the section of the steel beam gradually, along with the increase in height of the section of the steel beam. While the redistributed internal force of the concrete section reduces gradually, so does the total stress in the concrete slab. This indicates that the constraint of the steel beam to the creep of the concrete slab is more. The phenomenon above indicates that if the stiffness of the concrete keeps constant while the stiffness of the steel beam increases, the constraint of the steel beam to the creep of the concrete slab increases, the total sectional internal force of the steel beam increases, and the total sectional internal force of the concrete slab decreases. Because the total sectional internal force remains unchanged, the reduced internal force in the section of the concrete slab is transferred to the section of the steel beam.

The eighth column in Table 2 is the ratio of the redistributed bending moment of the section of the concrete slab to the full-sectional redistributed bending moment of the concrete slab section. As the sectional height of the steel beam increases gradually, the ratio becomes smaller gradually while the influence of redistributed bending moment of the section of the concrete slab on the axial deformation is also getting smaller and smaller. The ratio of the fifth section is only 1.9%, which is neglected in the simplified method and is very close to the ratio obtained with the exact method. Refer to the 5th to 8th sections in Table 2.

(15) $$\begin{array}{c} w_{s0}=\iint \frac{M_{s0}}{E_{s}I_{s}}dx^{2},\\ w_{st}=\iint \frac{M_{st}}{E_{s}I_{s}}dx^{2},\\ \frac{w_{st}}{w_{s0}}=\frac{M_{st}}{M_{s0}}. \end{array}$$

In the equation, *w*_*s*0_ and *w*_*st*_ are the deflections [25–27] of the steel beam before and after the creep. It can be seen from equation (13) that the stiffness of the steel beam is constant before and after the creep of the composite beam, and the deflection of the steel beam is proportional to the bending moment of the steel beam. The last column in Table 2 is ratios of bending moment of the steel beam before and after the creep. It can be seen that the deflection of the composite beam increases by 1.770–2.232 times, corresponding to the 1 ∼ 8 section, before and after the creep, when *φ*_*t*_=4 and *φ*_*f*,*d*_=2.57.

It can be seen intuitively from Figure 4 that *M*_*cr*_ and *N*_*cr*_ in the one concrete slab grows nonlinearly with fast speed (with large slope) in the area where the height of the steel beam is small, while they grow linearly with lower speed (with small slope) in the area where the height of the steel beam is large. *M*_*sr*_ is the redistribution of bending moment in the steel beam which is increasing linearly.

The axial direction and bending stiffness of steel beam and concrete slab will affect the redistribution of internal force of the section. In order to further investigate the changing regularity of the redistribution of internal force, this paper selects *α*_*cs*_ as the product ratio of two kinds of stiffness as the parameter to be investigated. Meanwhile, the method of comparing the precision and the simplified method are used to investigate errors of these two methods. The stress obtained by the calculation with the exact method and the simplified method is given in Table 3. Through comparison, it can be seen that the calculated errors of the two methods decrease with the decrease in *α*_*cs*_ which is the ratio of the axial direction of the concrete slab and the steel beam to the bending stiffness products of the concrete slab and the steel beam. The maximum error of two methods in the four edge stresses *σ*_*ct*_^*t*^, *σ*_*ct*_^*b*^, *σ*_*st*_^*t*^, and *σ*_*st*_^*b*^ with superscripts of *t* and *b* to indicate the top and bottom of the section, respectively, is the stress *σ*_*ct*_^*b*^ at the lower edge of the concrete slab. When *α*_*cs*_ ≤ 0.185, the maximum error is 1.027, less than 3%, at this time. The calculated result of the simplified method can fully meet requirements for the accuracy of calculation.

The analysis for data in Tables 2 and 3 is based on the premise of the constant creep coefficient to investigate the change regularity of the redistribution of internal force as the sectional height of the steel beam is changed. How will the internal force of the redistribution on the section of the steel beam and the concrete slab change if the height of the section of the steel beam is a fixed value under the conditions of the constant stiffness of the steel beam, the unchanged constraints to the concrete slab, and the change in creep coefficient? In this case, Section 6 that is shown in Table 1 is selected as the object of calculating analysis, and the creep coefficient is changed only. These changes are *φ*_*t*_ = 0, 1, 2, 3, 4, while the corresponding *φ*_*f*,*d*_ = 0, 0.43, 1.14, 1.86, 2.57. Results are shown in Table 4.

It can be seen in Table 4 that, as the creep coefficient increases, the redistribution of internal force increases while the axial force of concrete and steel beams decreases. Besides, the bending moment increases, especially the bending moment of steel beams. And the deflection after creep is 1.685–2.069 times than that before the creep. This shows the same phenomenon as increasing the height of the section of the steel beam. It shows the same phenomenon as that happening when the sectional height of the steel beam increases. This phenomenon indicates that there are two major factors affecting the redistribution of internal force, which are the stiffness of the steel beam (to constrain the creep stiffness) and the creep coefficient.

## 6. Conclusion

Rusch's exact approach and the simplified approach to solving the problem of the redistribution of the shrinkage and creep internal force of composite beam are analyzed and derived in this paper. After eight examples are elected for the calculation and analysis, three conclusions are obtained as the following:

1. Rusch's exact method is used to solve the problem of the redistribution of shrinkage and creep internal force of composite beams, and it is necessary to solve the coupled differential equations [28–30]. The volume of calculation is large with the complicated process. So, the practical applications are inconvenient and limited. The simplified method can be used to simplify the coupled differential equations into two independent differential equations with the simple process and simple calculated results. The error between the exact solution and the approximate solution shrinks as the parameter decreases. When *α*_*cs*_ ≤ 0.185, the error between the two is already small, within 3%, which can meet requirements for the accuracy of calculation. In addition, the ratio of the stiffness product [31] of the concrete slab to that of the steel beam in most composite beams is consistent, especially in the composite beam in the bridge structure, and the sectional height and stiffness of the steel beam are great.
2. Compared to the stiffness of the concrete slab, the greater the stiffness of the steel beam is, the more the constraints on the concrete slab are and the greater the redistribution of internal force caused by the shrinkage and the creep are. In other words, the stronger the final internal force of the steel beam is, the weaker the final internal force of the slab is.
3. If the stiffness of the steel beam and the concrete slab is constant, the larger the creep coefficient is, the greater the redistribution of internal force caused by the creep is. It means that the axial force of the concrete slab and the steel beam becomes smaller while the bending moment becomes larger, especially with the significant increase of steel beam. In addition, the increase in the stress of lower edge of the steel beam along with the change of creep coefficient is much smaller than that of the upper edge, which does not benefit the stability of the steel beam. Therefore, it should be paid attention to in engineering practice.
4. The premise of the simplified method in this paper is that the flexural stiffness of the concrete slab is obviously smaller than that of the steel beam, and the redistributed bending moment of the concrete slab will be relatively small. If the stiffness of the concrete slab is close to that of the steel beam, the redistributed bending moment is large and cannot be ignored, and this method is no longer applicable.

## Figures and Tables

**Figure 1:** (a) Dischinger's creep coefficient. (b) Rusch's creep coefficient.

**Figure 2:** The initial internal force and the redistribution of internal force of the section at the moment of *t*_0_, *t*, and *dt*.

**Figure 3:** Composite beam section.

**Figure 4:** The redistribution of inner force of the section under the variation of the height of steel beam.

**Table 1:** Detailed parameters of eight sections.

Sections	*h*_*s*_ (cm)	*A*_*cr*_ (cm^2^)	*I*_*cr*_ (cm^4^)	*A*_*s*_ (cm^2^)	*I*_*s*_ (cm^4^)	*A*_*i*_ (cm^2^)	*I*_*i*_ (cm^4^)	*S*_*i*_ (cm^3^)	*α*_*s*_=*A*_*s*_*I*_*s*_/*A*_*i*_*I*_*i*_	*α*_*c*_=*A*_*cr*_*I*_*cr*_/*A*_*i*_*I*_*i*_	*α*_*cs*_=*A*_*cr*_*I*_*cr*_/*A*_*s*_*I*_*s*_
1	40	816.3	27210.9	300.8	71261.3	1117.1	416583.2	836.2	0.046	0.048	1.036
2	60	816.3	27210.9	324.8	179012.0	1141.1	826907.0	1200.9	0.062	0.024	0.382
3	80	816.3	27210.9	348.8	344291.3	1165.1	1398481.2	1584.2	0.074	0.014	0.185
4	100	816.3	27210.9	372.8	573334.4	1189.1	2140161.0	1985.0	0.084	0.009	0.104
5	120	816.3	27210.9	396.8	872029.5	1213.1	3060480.9	2402.2	0.093	0.006	0.064
6	140	816.3	27210.9	420.8	1246016.2	1237.1	4167685.4	2835.0	0.102	0.004	0.042
7	160	816.3	27210.9	444.8	1700753.1	1261.1	5469756.7	3282.3	0.110	0.003	0.029
8	180	816.3	27210.9	468.8	2241563.9	1285.1	6974439.6	3743.4	0.117	0.002	0.021

**Table 2:** Internal forces of cross section (exact and approximate method).

Section	Initial internal force (*t*=0 and *φ*_*t*_=0)			Redistributed internal forces (*t*=*t* and *φ*_*f*,*d*_=2.57)			*M*_*cr*_/*M*_*cr*_+*M*_*sr*_	Final internal force = initial internal force + Redistributed internal forces			*M*_*st*_/*M*_*s*0_
	*N*_*c*0_	*M*_*c*0_	*M*_*s*0_	*N*_*cr*_	*M*_*cr*_	*M*_*sr*_		*N*_*ct*_	*M*_*ct*_	*M*_*st*_	
1	−4014.55	130.64	342.12	466.99 (636.49)	−85.94 (−80.52)	263.59 (322.66)	−0.484 (−0.333)	−3547.56 (−3378.06)	44.70 (50.12)	605.72 (664.78)	1.770 (1.943)
2	−2904.57	65.81	432.97	582.95 (640.43)	−42.72 (−41.77)	344.02 (372.78)	−0.142 (−0.126)	−2321.62 (−2264.14)	23.09 (24.04)	776.98 (805.75)	1.795 (1.861)
3	−2265.62	38.91	492.38	607.57 (632.50)	−24.55 (−24.28)	418.41 (434.31)	−0.062 (−0.059)	−1658.05 (−1633.12)	14.37 (14.63)	910.79 (926.69)	1.850 (1.882)
4	−1855.01	25.43	535.79	613.85 (626.43)	−15.47 (−15.38)	491.59 (501.25)	−0.032 (−0.032)	−1241.16 (−1228.58)	9.96 (10.05)	1027.37 (1037.04)	1.918 (1.936)
5	−1569.84	17.78	569.86	616.54 (623.57)	−10.39 (−10.35)	565.08 (571.36)	−0.019 (−0.018)	−953.30 (−946.28)	7.39 (7.43)	1134.95 (1141.23)	1.992 (2.003)
6	−1360.45	13.06	597.94	619.19 (623.40)	−7.30 (−7.28)	639.48 (643.77)	−0.012 (−0.011)	−741.26 (−737.04)	5.76 (5.78)	1237.42 (1241.71)	2.069 (2.077)
7	−1200.15	9.95	621.88	622.57 (625.24)	−5.30 (−5.29)	715.04 (718.07)	−0.007 (−0.007)	−577.58 (−574.91)	4.64 (4.66)	1336.91 (1339.95)	2.150 (2.155)
8	−1073.46	7.80	642.79	626.77 (628.53)	−3.95 (−3.95)	791.85 (794.06)	−0.005 (−0.005)	−446.68 (−444.92)	3.85 (3.85)	1434.64 (1436.85)	2.232 (2.235)

*Note*. The values in parentheses are obtained through the simplified method. Units of axial force and bending moment are kN and kNm, respectively.

**Table 3:** Stresses of cross section (precise and approximate method).

section	*α*_*cs*_=*A*_*cr*_*I*_*cr*_/*A*_*s*_*I*_*s*_	*σ*_*ct*_^*t*^ (N/mm^2^)	Precise/approximate	*σ*_*ct*_^*b*^ (N/mm^2^)	Precise/approximate	*σ*_*st*_^*t*^ (N/mm^2^)	Precise/approximate	*σ*_*st*_^*b*^ (N/mm^2^)	Precise/approximate
1	1.036	−6.11 (−6.10)	1.001	−2.76 (−2.34)	1.177	−238.24 (−261.49)	0.911	101.76 (111.66)	0.911
2	0.382	−3.77 (−3.73)	1.010	−2.04 (−1.93)	1.056	−180.86 (−187.56)	0.964	79.57 (82.51)	0.964
3	0.185	−2.61 (−2.59)	1.008	−1.53 (−1.49)	1.027	−144.99 (−147.52)	0.983	66.64 (67.81)	0.983
4	0.104	−1.92 (−1.91)	1.006	−1.18 (−1.16)	1.017	−121.03 (−122.17)	0.991	58.16 (58.71)	0.991
5	0.064	−1.47 (−1.46)	1.005	−0.91 (−0.90)	1.011	−104.05 (−104.63)	0.994	52.13 (52.41)	0.995
6	0.042	−1.14 (−1.14)	1.004	−0.71 (−0.70)	1.009	−91.45 (−91.76)	0.997	47.59 (47.75)	0.997
7	0.029	−0.90 (−0.89)	1.003	−0.55 (−0.54)	1.007	−81.74 (−81.92)	0.998	44.03 (44.13)	0.998
8	0.021	−0.70 (−0.70)	1.003	−0.41 (−0.41)	1.006	−74.04 (−74.16)	0.998	41.16 (41.22)	0.998

*Note*. Values in parentheses are results made by the simplified method. *σ*_*ct*_^*t*^, *σ*_*ct*_^*b*^ and *σ*_*st*_^*t*^, *σ*_*st*_^*b*^ are stresses of the upper and lower edges of the concrete slab and the steel beam, respectively.

**Table 4:** Stresses and internal forces of cross section.

Section internal force	Creep coefficient				
	*φ*_*t*_=0 and *φ*_*f*,*d*_=0	*φ*_*t*_=1 and *φ*_*f*,*d*_=0.43	*φ*_*t*_=2 and *φ*_*f*,*d*_=1.14	*φ*_*t*_=3 and *φ*_*f*,*d*_=1.86	*φ*_*t*_=4 and *φ*_*f*,*d*_=2.57
*N*_*c*0_ (kN)	−1398.7	−1360.45	−1360.45	−1360.45	−1360.45
*N*_*cr*_ (kN)	0.00	403.57	479.76	551.76	619.19
*N*_*ct*_ (kN)	−1398.70	−956.88	−880.69	−808.69	−741.26
*N*_*st*_ (kN)	1398.70	956.88	880.69	808.69	741.26
*M*_*c*0_ (kNm)	17.00	13.06	13.06	13.06	13.06
*M*_*cr*_ (kNm)	0.00	2.71	−2.56	−5.53	−7.30
*M*_*ct*_ (kNm)	17.00	15.77	10.50	7.53	5.76
*M*_*s*0_ (kNm)	555.00	597.94	597.94	597.94	597.94
*M*_*sr*_ (kNm)	0.00	409.33	492.38	568.87	639.48
*M*_*st*_ (kNm)	555.00	1007.27	1090.32	1166.81	1237.42
*M*_*st*_/*M*_*s*0_	1.000	1.685	1.823	1.951	2.069
*σ*_*ct*_^*t*^ (N/mm^2^)	−2.39	−1.79	−1.49	−1.29	−1.14
*σ*_*ct*_^*b*^ (N/mm^2^)	−1.11	−0.60	−0.71	−0.73	−0.71
*σ*_*st*_^*t*^ (N/mm^2^)	−40.99	−74.43	−80.57	−86.23	−91.45
*σ*_*st*_^*b*^ (N/mm^2^)	21.37	38.75	41.94	44.88	47.59

## Data Availability

The data used to support the findings of this study are available from the corresponding author upon request.
